# Adoption of Magnetic Resonance Image Features under Segmentation Algorithm in Effect Evaluation of Ginkgo Diterpenoid Lactone Glucamine Injection in Treatment of Cerebral Infarction

This article has been retracted.

**DOI:** 10.1155/2022/4558702

**Published:** 2022-04-15

**Authors:** Aidi Lei, Yanbo Zhang, Fulong Liang, Jianli Zhang, Jinle Cai

**Affiliations:** ^1^Department of Neurology, The Fifth Hospital of Xiamen, Xiamen 361101, Fujian, China; ^2^Department of Neurology, The Second Affiliated Hospital of Shandong First Medical University, Taian 271000, Shandong, China

## Abstract

Magnetic resonance imaging (MRI) image segmentation based on a segmentation algorithm was performed to assess neurological function in patients with acute cerebral infarction, to investigate the efficacy evaluation of Ginkgo diterpene lactones meglumine injection (GDLI) in the treatment of cerebral infarction and the efficiency of MRI image segmentation algorithm. First, the results of the fast semisupervised segmentation algorithm (algorithm group) and traditional processing (control group) were compared and analyzed. The recall rate, accuracy, recognition accuracy, and segmentation time of the two groups were compared. The control group was given conventional treatment, while the algorithm group was given GDLI based on conventional treatment. Finally, the difference in serum vascular endothelial growth factor (VEGF), hypoxia-inducible factor-la (HIF-la), angiotensin (Ang)-1, Ang-2, and interleukin (IL)-6 protein concentration was analyzed after treatment. The algorithm evaluation results showed that the accuracy and recall rate of MRI images recognized by the algorithm group fluctuate at 90%. In the control group, the accuracy and recall rate of MRI image results fluctuated at 80%, and the data were statistically different (*p* < 0.05). The clinical index test results showed that the serum VEGF content of the test group was higher than that of the control group, and the data was statistically different (*p* < 0.05). In addition, the cerebral blood flow (CBF) and cerebral blood volume (CBV) of the lesion side of the algorithm group were greatly higher than those of the control group on the 30th day, and the differences were significant (*p* < 0.05). There was little difference between the method presented in this study and the manual delineation by a physician. Compared with traditional manual segmentation, this method greatly reduced the time required for the segmentation of lesions. The diagnostic specificity, sensitivity, and accuracy of the images segmented by the fast semisupervised algorithm were higher than those of the conventional method, and the diagnostic accuracy of acute cerebral infarction was high. In addition, it was sensitive and accurate to detect acute cerebral infarction, which provided a reliable reference for early diagnosis and condition judgment of patients.

## 1. Introduction 

Cerebral infarction is an acute cerebral vascular disorder characterized by high mortality, high recurrence rate, and many complications. It is one of the main diseases leading to human death, and the incidence of cerebral infarction is increasing year by year [1]. The main cause of cerebral infarction is the irreversible injury of brain tissue and cells caused by intracranial vascular occlusion. The severity of cerebral infarction lesion depends on various factors such as cerebral ischemia site, lateral blood circulation path, and arterial root lesion. Early monitoring and treatment are effective methods to reduce the recurrence rate and mortality of cerebral infarction [2]. Chemical agents exert their efficacy mainly through the control of personal signs such as blood pressure, blood glucose, and blood lipids [3]. Acting on multiple targets, TCM injections are characterized by rapid absorption and high bioavailability and play an increasingly important role in the prevention and treatment of acute and severe clinical diseases [4]. Ginkgolide compounds belong to terpenoids, also known as ginkgolide lactones, and are an important active component in *Ginkgo biloba* leaves [5, 6].

The flavonoids of *Ginkgo biloba* leaves have the ability to remove free radicals, so they can accelerate the repair of damaged neurons and play a role in protecting brain nerves in case of brain damage [7]. The 6-hydroxyphosphoric acid of *Ginkgo biloba* leaves can inhibit the toxic damage caused by irritating amino acids, so it has the effect of protecting nerve cells [8]. At present, the traditional morphological imaging method is still difficult to evaluate the heterogeneous lesions of different types of acute cerebral infarction, and the quantitative value of the lesions is difficult to visualize [9]. Therefore, it is important to assess the extent of cerebral infarction lesions and to predict the pathological and physiological status of the ischemic region for clinical treatment decisions.

Imaging optics are helpful to reflect the pathological characteristics of some morphological properties [10]. Image segmentation is a part of artificial intelligence, which is defined as the data extraction and mining of medical images in the field of medical images. Multiple image segmentation analysis features such as size, shape, and texture are obtained, which reflect the subtle features within the image and are used for large-scale image information analysis [11]. Artificial intelligence image segmentation is used for quantitative evaluation of lesions, for it can reflect the focal points of lesions [12]. At present, magnetic resonance imaging (MRI) has been widely used in the field of clinical diagnosis and has shown high application value in the examination of cerebral infarction. This technique is not easily affected by bone artifacts and has high accuracy in diagnosis. Based on these results, it can accurately understand the craniocerebral anatomical structure of patients and provide support for the formulation of the appropriate treatment plan. In the diagnosis of cerebral infarction, MRI can accurately distinguish lesions and surrounding tissues, and the corresponding diagnostic sensitivity is significantly improved, which lays a good foundation for reducing the rate of missed diagnosis. The advantages of MRI include high accuracy of structure judgment and diagnosis, which is free from artifact interference. It can effectively detect early cerebral infarction with high differentiation. It can accurately detect early cerebral infarction and has obvious advantages in diagnosing cerebral stem infarction. Despite the high performance, high efficiency, and fast performance of many medical image technologies, MRI technology as an auxiliary method of brain image is very popular in the clinical diagnosis of brain diseases [13]. However, MRI images are still affected by motion artifacts and noise due to the irregularity of MRI motion, the complex structure of brain physiology, and tissue blur. Moreover, cerebral infarction is characterized by diversity and brain artifacts [14].

To solve these problems, the segmentation algorithm for MRI images of cerebral vascular infarction lesions was discussed. To solve the problems of traditional doctors' judgment errors and excessive time-consuming, an improved local constrained sfokes-FCM algorithm was proposed. In brain MRI images, the adaptive segmented brain algorithm had strong antinoise performance, strong strength, and accuracy according to the location, area, and brain tissue of the lesion. It can distinguish lesions from brain MRI images, improve image accuracy, and shorten diagnosis time. Ginkgo diterpene lactones meglumine injection (GDLI) was used to treat patients with cerebral infarction, and the treatment effect was analyzed from multiple indicators.

## 2. Methods

### 2.1. Research Objects

Patients were selected from 80 patients in the hospital from June 2018 to December 2019. According to the inclusion and exclusion criteria, 60 patients meeting the criteria were selected and randomly rolled into two groups (each group with thirty subjects). The GDLI treatment group was analyzed using algorithms (algorithm group), and the GDLI treatment group (control group) was analyzed using MRI images by traditional physicians. In this study, a total of 60 patients with acute cerebral infarction met the inclusion criteria and exclusion criteria. This study had been approved by the Medical Ethics Committee of the Hospital, and all the families of the patients included in the study had signed the informed consent.

#### 2.1.1. Inclusion Criteria

Inclusion criteria were as follows: (a) the patient had cerebral infarction demonstrated by intracranial CT; (b) the patient had acute brain lesions within 72 hours confirmed by MRI; (c) the patient had acute cerebral infarction; (d) the patient had a history of cerebral infarction but had not been cured, and the patient was still under observation and treatment in the inpatient department.

#### 2.1.2. Exclusion Criteria

Exclusion criteria were as follows: (a) patients with intracerebral hemorrhage, (b) patients with transient cerebral ischemia, (c) other brain diseases, (d) patients with systemic neurological disease, (e) severe liver dysfunction, (f) pregnant, breastfeeding, or planned pregnancy, and (g) patients under 25 years of age.

### 2.2. Principle of Fast Semisupervised Algorithm

Semifuzzy fast C-means (SFFCM) is a new algorithm structure created by combining the advantages of fast generalized fuzzy C-means (FGFCM) and semifuzzy C-means (s FCM) semisupervised FCM algorithms.

According to the characteristics of the lesion in the MRI image of cerebral infarction, the appropriate starting number and coordinate points centered on the threshold are set, and the threshold processing sometimes brings very different results. It needs to be adjusted at any time when the parameters are set, and the result of the algorithm will be more accurate. In addition, in terms of the number of functions such as the position, area, and settings of the MRI image, the function is mainly determined according to the location of the lesion. To reduce the value deviation of the objective function as much as possible, multiple adjustments and calculations are required. The SFFCM algorithm equation is as follows.

(1) $$\begin{array}{c} J=\overset{C}{\underset{i=1}{\sum }}\overset{N}{\underset{k=1}{\sum }}\mu_{ik}^{m}{\left\|y_{k}|-|b_{k}|-|v_{i}\right\|}^{2}+\alpha \overset{C}{\underset{i=1}{\sum }}\overset{N}{\underset{k=1}{\sum }}f_{ik}^{-1}u_{ik}^{m}{\left\|\overset{¯}{y_{k}}|-|b_{k}|-|v_{i}\right\|}^{2}. \end{array}$$

In this algorithm, *b*_*k*_ represents the partial constraint value of the average neighboring pixels of the *k*th pixel, and *f*_*ik*_^−1^ represents the probability function of the average neighboring pixels of the *k*th pixel. When the equation is calculated, the value range of *f*_*ik*_^−1^ is 0–1. This equation yields a fuzzy membership function.

(2) $$\begin{array}{c} \mu_{ik}=\frac{1}{\sum_{i=1}^{C}\left(\left\|y_{k}-b_{k}-v_{i}\right\|/{\left.\left\|y_{k}-b_{k}-v_{i}\right\|\right)}^{1/m-1}\right.}. \end{array}$$

This equation gives the local membership function as follows.

(3) $$\begin{array}{c} U_{ik}=\frac{\left(f_{ik}\right)1/m-1}{\sum_{i=1}^{C}{\left(f_{ik}\left\|\bar{y_{k}}-b_{k}-v_{i}\right\|/\left\|y_{k}-b_{k}-v_{l}\right\|\right)}^{1/m-1}}. \end{array}$$

The equation for recalculating cluster centers is as follows:

(4) $$\begin{array}{c} v_{i}=\frac{\sum_{k=1}^{N}\left(\mu_{ik}^{m}\left(y_{k}-b_{k}\right)+\alpha f_{ik}^{-1}u_{ik}^{m}\left(\overset{¯}{y_{k}}-b_{k}\right)\right)}{\sum_{k=1}^{N}\left(\mu_{ik}^{m}-\alpha f_{ik}^{-1}u_{ik}^{m}\right)}. \end{array}$$

The above three equations are integrated to obtain the joint membership function as follows:

(5) $$\begin{array}{c} z_{ik}=\frac{{\left(\mu_{ik}\right)}^{p}{\left(u_{ik}\right)}^{q}}{\sum_{c=1}^{C}{\left(\mu_{ck}\right)}^{p}{\left(u_{ck}\right)}^{q}}. \end{array}$$

The joint clustering center equation is as follows.

(6) $$\begin{array}{c} w_{i}=\frac{\sum_{k=1}^{N}Z_{ik}^{m}\left(y_{k}-b_{k}\right)}{\sum_{k=1}^{N}z_{ik}^{m}}. \end{array}$$

The joint membership function integrates the aggregation class center equation as follows:

(7) $$\begin{array}{c} J^{\prime }=\sum_{i=1}^{C}\sum_{k=1}^{N}z_{ik}^{m}{\left(y_{k}-b_{k}-w_{i}\right)}^{2}. \end{array}$$

The joint membership function integrates the derivation of the aggregate class center to obtain the new neighborhood local constraint value expression as follows:

(8) $$\begin{array}{c} b_{k}=y_{k}-\frac{\sum_{i=1}^{C}z_{ik}^{m}w_{i}}{\sum_{i=1}^{C}z_{ik}^{m}}. \end{array}$$

After the value is substituted, it is compared with the preset threshold to calculate the new cluster center value and a new local limit value needs to be calculated, to change the original value and reset the judgment condition of the operation. The new cluster center value is calculated repeatedly, and if the new value is less than the original value, the lesion location is segmented or cyclically operated.

### 2.3. Algorithm Specific Process

The objective function is further integrated, and the local gray area statistics method is added. The relationship between the number of pixels and the neighboring pixels is combined. For the setting of the threshold, the number of clusters, the initial cluster center, and the initial value, it is necessary to consider the MRI image of the cerebral vascular infarction that should be recognized. It needs to fully consider the difference between large lesions and small lesions. In the case of large lesions, it is necessary to completely segment the lesions while considering the effects of artifacts in specific MRI images.

The segmentation process of the SFFCM algorithm for cerebral infarction is as follows. (a) Input MRI image of the ischemic site of cerebral infarction. (b) Make local location statistics. (c) Initialize parameters and initialize the aggregation center. (d) Calculate local membership degree according to the equation. (e) Update the joint membership degree. (f) Determine pixel attribution according to membership degree. (g) Output location of lesion analysis. The specific algorithm flow is shown in Figure 1.

### 2.4. Detection of Serum VEGF, HIF-La, Ang-1, Ang-2, and IL-6 Protein Concentration by Enzyme-Linked Immunoassay

The control group received conventional treatment, while the algorithm group received an intravenous infusion of GDLI once a day (30 mL) based on conventional treatment. The indexes were measured at one day, two weeks, and one month after treatment.

Within one day and on the 30th day after the patient was admitted to the hospital, a head MRI was performed to detect the patient's cerebrovascular condition. One day, two weeks, and one month after the patient's admission, 2.5 mL of cubital vein serum was collected on an empty stomach in the early morning, placed at room temperature for one hour, and centrifuged at 3, 000 r/min for 10 minutes. Then, the serum was separated and stored in a refrigerator at −80°C for later use. Enzyme-linked immunoassay was adopted to detect serum vascular endothelial growth factor (VEGF), hypoxia-inducible factor-la (HIF-la), angiotensin (Ang)-1, Ang-2, and interleukin (IL)-6 protein concentration.

Samples included serum of patients to be tested. Reagents included HRP-conjugate antibody (anti-HBS), HBsAg positive control serum, negative control, washing solution, chromogenic agents A and B, and termination solution. Equipment included microreaction plate (48 well) coated with antibody, micropipette, and microplate reader. The procedure of ELISA was as follows. (a) 50 *μ*L sample was added to each well of microreaction plate, two wells each were set as positive and negative controls, one drop of positive (or negative) control was added to each well, and one well of blank control was set. (b) One drop of enzyme binder was added to each well (except blank control) and mixed well, and the plate was sealed and incubated at 37°C for 30 minutes. (c) The liquid in the wells was discarded, and the wells were filled with washing liquid, standing for five seconds, dried, repeated five times, and dried. (d) One drop of chromogenic solution A and one drop of chromogenic solution B were added to each well and mixed well, and the plate was sealed and incubated at 37°C for 15 minutes. (e) One drop of termination solution was added to each well and mixed well. (f) A microplate reader performed the reading, the wavelength of 450 nm was taken, the blank hole was measured and adjusted to zero first, and then the OD value of each well was read.

### 2.5. Magnetic Resonance Scanning Process

Image acquisition required that all patients underwent a 3.0 TMR scan. The matching 12 channel head coil was utilized. The patient was placed in a supine position with matching earphones to reduce noise stimulation. The matching sponge pad was placed between the subject's head and the MR coil to reduce the subject's head movement. Subjects underwent routine MRI examinations at axial T2WI, axial T1WI, and sagittal position. After the nature, size, and location of the lesion were determined by conventional MRI, the largest layer of the lesion was selected for scanning. Subsequently, all patients underwent a head CT scan or/and SWI under the MR system to confirm or rule out cerebral hemorrhage.

### 2.6. Data Processing and Analysis

MATLAB was used to process image data. The fast Fourier transform of frequency domain analysis method was adopted to transform MRI images from the time domain to the frequency domain, which was convenient to extract and analyze image features. After a fast Fourier transform, real fraction mapping, virtual fraction mapping, and phase component mapping of MRI images were generated. The differential diagnosis of acute ischemic stroke and acute cerebral hemorrhage was performed by using real part mapping of MRI images.

### 2.7. Statistical Methods

All experimental statistics were statistically analyzed using SPSS 20.0. The data all obeyed the normal distribution, and the related measurement data were all expressed by the mean ± standard deviation ($\bar{\text{x}}$ ± *s*). The comparisons before and after treatment in the data group were all carried out by paired *t*-test, and all were carried out by one-way analysis of variance. *p* < 0.05 indicated that the difference was substantial.

## 3. Results

### 3.1. Comparison of Cerebral Infarction Lesions Segmented by SFFCM Algorithm and Traditional Physicians

The visual assessment method was used to compare the results of neurocerebral infarction infarcts manually segmented by the method and the doctor, as shown in Figures 2(a) and 2(b). On MRI images, using algorithms to segment infarcts was relatively more accurate, and the number of identified lesions was close to that of physicians' manual segmentation, indicating that the overall effect of algorithm recognition was excellent.

Measuring the accuracy and recall of the two methods can intuitively analyze the image segmentation effect, as shown in Figure 3. The recognition result recall rate of the algorithm group fluctuated at 80–90%, and the recognition result recall rate of the control group fluctuated at 79–82%. The algorithm group had a greatly higher recall rate. In Figure 4, the algorithm group's recognition result accuracy rate fluctuated between 80 and 86%, and the control group's recognition result accuracy rate fluctuated between 65 and 72%. The algorithm group had a greatly higher accuracy rate, and the data was statistically different (*p* < 0.05).

Measuring the accuracy of the two methods in different parts can intuitively analyze the image segmentation effect. In Figure 5, for image recognition in the white matter range, the accuracy of the recognition results of the algorithm group fluctuated between 60 and 80%, and the accuracy of the control group's recognition results fluctuated between 44 and 65%. There were statistical differences in the data (*p* < 0.05). In Figure 6, when image recognition was performed in the gray matter range of the brain, the accuracy of the recognition results of the algorithm group fluctuated between 60 and 100%, and the accuracy of the recognition results of the control group fluctuated between 42 and 62%, with a statistical difference (*p* < 0.05). In Figure 7, when image recognition was performed in the range of the brain and spinal cord, the accuracy of the recognition results of the algorithm group fluctuated between 60 and 80%, and the accuracy of the recognition results of the control group fluctuated between 36 and 55%, with a statistical difference (*p* < 0.05).

The comprehensive comparison was implemented for algorithm-based MRI recognition methods of cerebral vascular infarction and traditional feature extraction methods to recognize cerebral vascular infarction. The algorithm proposed in this study was better than traditional feature extraction and recognition methods, and the results are shown in Figures 8 and 9. The correct recognition rate proposed by the algorithm group of this research was maintained at 58%, and the correct recognition rate proposed for the control group was maintained at 54%. The segmentation time of the algorithm group was 0.59 seconds/frame, and the segmentation time of the control group was 4.77 seconds/frame. Therefore, the proposed segmentation algorithm was of a certain effect on recognizing cerebral vascular infarction in MRI images.

### 3.2. Blood Test Result Indicators

The comparisons of the serum VEGF levels measured on the first day, two weeks, and one month of admission between the two groups of patients are shown in Figure 10. On the first day, the difference in content between the two groups was 125 (pg/mL), and the values were not statistically different (*p* > 0.05). After two weeks, the serum VEGF content in the algorithm group reached 1000 (pg/mL). Compared with the control group's serum VEGF content of 810 (pg/mL), the data was statistically different *p* < 0.05(*p* < 0.05). After one month of treatment, the data of the two groups were statistically different (*p* < 0.05).

The serum HIF-a content of the patient was detected, and the results are shown in Figure 11. On the first day, the content of the two groups differed by 233 (pg/mL), and the values were not statistically different (*p* > 0.05). Two weeks later, the serum HIF-a content in the algorithm group reached 640 (pg/mL), which was reduced by about 400 (pg/mL). Compared with the control group's serum HIF-a content of 570 (pg/mL), the data had statistical differences (*p* < 0.05). After one month of treatment, the two groups' data had statistical differences (*p* < 0.05).

The serum Ang-1 content of the patient was detected, and the results are shown in Figure 12. On the first day, the difference in content between the two groups was 7 (pg/mL), and the values were not statistically different (*p* > 0.05). Two weeks later, the serum Ang-1 content in the algorithm group reached 17.2 (pg/mL), which decreased by 11 (pg/mL). Compared with the control group's serum Ang-1 content of 12 (pg/mL), the data was statistically different (*p* < 0.05). After one month of treatment, the data of the two groups were statistically different (*p* < 0.05), suggesting that the adoption of the proposed algorithm was helpful to reduce the level of Ang-1 in serum.

The serum Ang-2 content of the patient was detected. The results are shown in Figure 13. The difference between the two groups on the first day was 5 (pg/mL), and the values were not statistically different (*p* > 0.05). Two weeks later, the serum Ang-2 content of the algorithm group reached 38.3 (pg/mL). Compared with the control group's serum Ang-2 content of 32.6 (pg/mL), the data was statistically different (*p* < 0.05). After one month of treatment, the data of the two groups were statistically different (*p* < 0.05), suggesting that the adoption of the proposed algorithm was helpful to increase the content of Ang-2 in the serum.

The serum IL-6 content of the patient was detected. The results are shown in Figure 14. The difference between the two groups on the first day was 9 (pg/mL), and the values were not statistically different (*p* > 0.05). Two weeks later, the serum IL-6 content of the algorithm group reached 56.38 (pg/mL). Compared with the control group's serum IL-6 content of 64.24 (pg/mL), the data was statistically different (*p* < 0.05). After one month of treatment, the data of the two groups were statistically different (*p* < 0.05), suggesting that the adoption of the proposed algorithm was helpful to increase the IL-6 content in serum.

### 3.3. Comparison of Imaging Indicators between the Two Groups

The comparisons of cerebral blood flow (CBF) and cerebral blood volume (CBV) before and after the lesion on the 30th day and the 1st day between the algorithm group and the control group are shown in Figures 15 and 16. On the 30th day, the CBF content was 38.2 (mL/100 g/min), and the CBF content of the control group was 36 (mL/100 g/min). The difference was substantial (*p* < 0.05). Compared with the control group, the CBF and CBV on the affected side of the algorithm group showed increased blood flow and blood volume. The difference was substantial (*p* < 0.05).

Comparisons of the TTP and MTT time values of the affected side on the 30th day and the 1st day between the algorithm group and the control group are shown in Figures 17 and 18. On the first day of treatment, there was no substantial difference in the TTP and MTT time values of the affected side of the two groups of patients (*p* > 0.05). After 30 days of treatment, the TTP and MTT time values of the affected side of the algorithm group were shortened compared with those of the control group, indicating that the blood passing time increased faster than before, and the difference was substantial (*p* < 0.05).

## 4. Discussion

Acute cerebral infarction is a common multiple disease in clinics. There are cerebral tissue necroses after the sharp interruption of blood flow in the cerebrovascular system [15]. The incidence of acute cerebral infarction is sharp, the disease develops rapidly, the neurological function of patients is impaired, and the mortality rate is high, which causes different degrees of damage. Active treatment of clinical acute cerebral infarction is the key to treatment [16]. Because of the particularity of brain anatomy and brain tissue, the diagnosis of acute cerebral infarction by neurographic examination occupies an important position. MRI can map different brain structures with clear images and high soft tissue resolution [17, 18]. Although previous MRI scans are used to show the lesions of acute cerebral infarction, previous MRI plane scans also have poor diagnosis or misdiagnosis [19].

Studies revealed that cerebral ischemia spreads within two hours of cerebral ischemia with underdiagnosed cytotoxic edema following vasogenic edema following cerebral ischemia. After the response of the ischemic region to water molecules is altered by using diffuse-sensitive gradient fields, due to the ischemic response of brain tissue in patients with acute cerebral infarction, cerebral blood flow is insufficient, and this feature is shown as a high signal. In this study, the diagnostic sensitivity, specificity, and accuracy of AI-segmented MRI images were higher than those of previous MRI images (*p* < 0.05), referring to clinical comprehensive diagnosis results. The serum HIF-a content of patients was detected. After two weeks, the serum HIF-a content of the algorithm group reached 640 (pg/mL), decreased by about 400 (pg/mL). Comparison of focal-side cerebral blood flow (CBF) and cerebral blood volume (CBV) between the experimental group and the control group on day 30 and day 1 showed that CBF content on day 30 was 38.2 (mL/100 g/min), while CBF content in the control group was 36 (mL/100 g/min); the differences were statistically significant (*p* < 0.05). Compared with the control group, CBF and CBV of the affected side of the experimental group increased, and blood flow and volume recovered, which was similar to the results of Frank et al. [20]. It indicated that AI-segmented MRI images had a good coincidence between the diagnosis results of acute cerebral infarction and clinical comprehensive diagnosis results. The coincidence between MRI and clinical comprehensive diagnosis was not good in the past. The consistency between conventional MRI and clinical comprehensive diagnosis results was only moderate, indicating that the diagnostic accuracy of AI-segmented MRI images for acute cerebral infarction was better than that of conventional MRI.

## 5. Conclusion

This study showed that after MRI images were used during the treatment of acute cerebral infarction with GDLI, there was little difference between the proposed method and the physician's manual delineation of the infarct area on the MRI image, whether using the subjective or objective assessment methods. Compared with traditional manual segmentation, this method greatly reduced the time required for the segmentation of lesions. Moreover, the diagnostic specificity, sensitivity, and accuracy of AI segmentation images were higher than those of conventional MRI (*p* < 0.05), and the diagnostic accuracy of AI segmentation images was higher than that of conventional MRI (*p* < 0.05). It was sensitive and accurate to detect acute cerebral infarction, which provided a reliable reference for early diagnosis and condition judgment of patients.

## Figures and Tables

**Figure 1:** SFFCM algorithm segmentation flow chart of cerebral infarction.

**Figure 2:** Comparison of MRI infarct segmentation. (a) Manual segmentation by the physician; (b) algorithm segmentation.

**Figure 3:** Comparison of recognition recall rates between the two groups.

**Figure 4:** Comparison of the accuracy of recognizing images between the two groups.

**Figure 5:** Comparison of the recognition accuracy of the white matter image range between the two groups.

**Figure 6:** Comparison of the recognition accuracy of the two groups of brain gray matter image ranges.

**Figure 7:** Comparison of the accuracy of the range recognition of the two groups of the brain and spinal cord images.

**Figure 8:** Comparison of the correct recognition rate of the segmentation algorithm and traditional feature extraction to identify cerebral vascular infarction. ^*∗*^*p* < 0.05.

**Figure 9:** Comparison of segmentation time comparison between segmentation algorithm and traditional feature extraction to identify cerebral vascular infarction. ^*∗*^*p* < 0.05.

**Figure 10:** The serum VEGF levels of the two groups of patients in one day, two weeks, and one month. ^*∗*^Compared with the control group, *p* < 0.05.

**Figure 11:** Serum HIF-a levels of the two groups of patients in one day, two weeks, and one month. ^*∗*^Compared with the control group, *p* < 0.05.

**Figure 12:** Serum Ang-1 levels of the two groups of patients in one day, two weeks, and one month. ^*∗*^Compared with the control group, *p* < 0.05.

**Figure 13:** The levels of serum Ang-1 in the two groups of patients in one day, two weeks, and one month. ^*∗*^Compared with the control group, *p* > 0.05.

**Figure 14:** The levels of serum IL-6 in the two groups of patients in one day, two weeks, and one month. ^*∗*^Compared with the control group, *p* < 0.05.

**Figure 15:** Comparison of CBF on the focal side of the two groups of patients on one day and one month. ^*∗*^Compared with the control group, *p* < 0.05.

**Figure 16:** Comparison of CBV on the focal side of the two groups of patients on one day and one month. ^*∗*^Compared with the control group, *p* < 0.05.

**Figure 17:** Comparison of TPP on the affected side of the two groups of patients on one day and one month. ^*∗*^Compared with the control group, *p* < 0.05.

**Figure 18:** Comparison of MTT on the affected side of the two groups of patients on one day and one month. ^*∗*^Compared with the control group, *p* < 0.05.

## Data Availability

The data used to support the findings of this study are available from the corresponding author upon request.
